# Biomedical Text Classification Using Augmented Word Representation Based on Distributional and Relational Contexts

**DOI:** 10.1155/2023/2989791

**Published:** 2023-02-15

**Authors:** Md. Aslam Parwez, Mohd. Fazil, Muhammad Arif, Md Tabrez Nafis, Md. Rabiul Auwul

**Affiliations:** ^1^Department of Computer Science & Engineering, Jamia Hamdard, New Delhi, India; ^2^University of Limerick, Limerick, Ireland; ^3^Department of Computer Science, Superior University Lahore, Lahore 54000, Pakistan; ^4^Department of Statistics, Bangabandhu Sheikh Mujibur Rahman Agricultural University, Gazipur 1706, Bangladesh

## Abstract

Due to the increasing use of information technologies by biomedical experts, researchers, public health agencies, and healthcare professionals, a large number of scientific literatures, clinical notes, and other structured and unstructured text resources are rapidly increasing and being stored in various data sources like PubMed. These massive text resources can be leveraged to extract valuable knowledge and insights using machine learning techniques. Recent advancement in neural network-based classification models has gained popularity which takes numeric vectors (*aka word representation*) of training data as the input to train classification models. Better the input vectors, more accurate would be the classification. Word representations are learned as the distribution of words in an embedding space, wherein each word has its vector and the semantically similar words based on the contexts appear nearby each other. However, such distributional word representations are incapable of encapsulating relational semantics between distant words. In the biomedical domain, *relation mining* is a well-studied problem which aims to extract relational words, which associates distant entities generally representing the subject and object of a sentence. Our goal is to capture the relational semantics information between distant words from a large corpus to learn enhanced word representation and employ the learned word representation for various natural language processing tasks such as text classification. In this article, we have proposed an application of biomedical relation triplets to learn word representation through incorporating relational semantic information within the distributional representation of words. In other words, the proposed approach aims to capture both distributional and relational contexts of the words to learn their numeric vectors from text corpus. We have also proposed an application of the learned word representations for text classification. The proposed approach is evaluated over multiple benchmark datasets, and the efficacy of the learned word representations is tested in terms of *word similarity* and *concept categorization* tasks. Our proposed approach provides better performance in comparison to the state-of-the-art GloVe model. Furthermore, we have applied the learned word representations to classify biomedical texts using four neural network-based classification models, and the classification accuracy further confirms the effectiveness of the learned word representations by our proposed approach.

## 1. Introduction

Biomedical literature, medical records, clinical notes, and online databases such as PubMed are the treasury of valuable information that is rapidly increasing in volume and size. Biomedical professionals and researchers are exploring and analyzing these large volumes of structured and unstructured texts to extract and curate valuable information using different knowledge discovery and data mining techniques. In this line, automated text classification using machine learning techniques has always been considered as a key technique to categorize, filter, search, manage, or process a large volume of text documents. Text classification is a key natural language processing (NLP) task wherein texts are labeled with specific classes based on their contents. Such labeling helps to extract valuable information for various applications, such as disease surveillance, information extraction, named-entity recognition, topic labeling, and social media monitoring.

In the biomedical domain, the existing literature is a valuable source of a large number of named entities, concepts, features, and their associations. In this domain, text classification has many applications including allocating medical subject headings (MeSH terms) to the biomedical articles [1, 2], identifying reportable disease cases from the clinical and pathological reports, and categorizing biomedical documents based on their content. Furthermore, classifying biomedical texts could help to improve the performance of gene-disease association extraction, protein-protein interaction extraction, understanding the functioning of genes, or discovering any other kind of knowledge. The efficiency and accuracy of any classification system depend on the classification algorithm (or the classifier) used and the input feature on which it operates. Since a classifier learns a model from the training data in the form of feature vectors, the role of feature vectors or feature representation is very important in classification performance. In NLP tasks, word representation (*aka* word embedding) has a notable influence on the performance of deep learning-based classification models.

### 1.1. Traditional Word Representation and Its Limitations

In traditional word representation techniques, words are encoded as vectors of binary, tf (term frequency), or tf-idf values, where tf-idf stands for “term frequency inverse-document frequency” that have yielded promising results for the classification task. These vectors consider lexical features such as uni-gram, bi-gram, or n-grams (*n* > 2) to represent text documents as feature vectors, with each entry of the vector consisting of either a Boolean value or frequency count to indicate the presence of lexical features. However, such vectors are unable to capture the semantic information because they ignore the context and the order of the words in the documents. Besides the problems of ignoring word order and contextual information, these feature vectors also suffer from data sparsity issues. Such issues have been addressed using neural network models to learn word representation as low-dimensional dense vectors.

### 1.2. Modern Word Representation and Its Limitations

Recently, the distributional representation of words as feature vectors (*aka words embedding*) has opened a new horizon in NLP applications because of its nature to capture contextual information and, hence, the semantics of words mentioned within the textual contents. Learning such word representations as low-dimensional dense vectors in an embedding space from a large corpus has gained popularity since the pioneering work of Mikolov et al. [3]. Such word vectors aim to capture the distributional features of words in a large corpus. Many NLP problems such as classification, clustering, and sentiment analysis have been solved by employing these word representations. Furthermore, the resurgence in the neural network-based machine learning algorithms has shown their capability to accomplish high accuracy even with less engineered features.

Towards this direction, Word2Vec [3] and GloVe [4] are two important algorithms that are widely used to learn distributional representation of words as low-dimensional dense vectors, which can be employed to enhance the performance of neural network-based classification systems. These algorithms consider the neighboring context words on either side of a target word within a fixed context window to preserve the distributional similarity of words. However, these distributional word representations have two major shortcomings: (i) They are inept in capturing relational semantics of words because of their dependence on fixed context window, and (ii) the rare co-occurrence of word pairs might be further problematic as a large corpus may not have a sufficient co-occurrence count of the rare word pairs. To eliminate these shortcomings, researchers tried to incorporate relational knowledge from third-party knowledge bases (KBs) such as WordNet [5] and Freebase [6] into the distributional representation of words. Semantic relations such as synonymy, hypernymy, and meronymy from the KBs have been incorporated into the distributional representation of words to learn better word representations [7, 8]. The relations from KBs, though rich in terms of semantic information, may have inadequate entries and also lack the contextual information. Furthermore, KBs are generally manually curated and maintained due to which they may not be comprehensive.

In addition, the existing works consider only linear contexts to derive contextual information of a target word, wherein context words are the surrounding words within the window of *k* tokens that precede and follow the target word. For example, in the sentence “Whipple disease is a rare systemic illness characterized by arthralgias, chronic diarrhea, weight loss, fever, and abdominal pain,” the words in the pair (*Whipple*, *fever*) or (*Whipple*, *pain*) have long-range association representing their relational semantics. Both *fever* and *pain* are semantically related to *Whipple* as they are symptoms of *Whipple* disease. These distant relationships will not be captured by a fixed context window of *k* = 5 or 10. The smaller context window, say, *k* = 2 may fail to capture important context, while a very large context window may capture weak and irrelevant contexts, resulting in an adverse impact on the embedding representation. In the existing literature, to capture the distributional context of words, the most commonly used context window size is *k* = 5. Additionally, if we aspire to learn word embeddings from domain-specific corpus, say, biomedical text corpus, then the semantic associations between *Whipple* disease and *fever* or *Whipple* disease and *pain* would be of extreme importance as *fever* and *abdominal pain* are symptoms of *Whipple* disease. Furthermore, the rare co-occurrence of such semantically associated words may have little or no weightage during their distributed representation, and it may fail to capture the semantics of such associations. Therefore, the inclusion of such relational information into the distributional representation will enrich and enhance the quality of word representation.

In addition to linear window-based bag-of-word contexts, the syntactic contexts have also been used to generate dependency-based word embeddings [9]. The syntactic contexts are the words that are linked with a target word through syntactic dependency relationships generated by a parser. These syntactic contexts can capture the functional similarity of words [9]. For example, the dependency graph of an example sentence produced by the Stanford parser is shown in Figure 1, which depicts the dependency relations on the edge labels of the graphs. Levy and Goldberg [9] used direct and inverse dependency relations for the target word to generate its dependency-based contexts to learn syntactic dependency-based word embedding. However, these dependency-based contexts with direct and inverse relations at one hop distance in the dependency graphs are unable to capture the semantics of words, which are at multihop (distant) dependency relations in the graph.

In biomedical literature, many traditional approaches for text classification exist; however, the recent popularity of deep learning models such as convolutional neural networks (CNNs) and long-short term memory (LSTM) has drawn the attention of researchers in the biomedical domain to achieve better performance in various NLP and text classification tasks. These deep learning models together with the word embeddings have shown remarkable performance in biomedical text classifications.

### 1.3. Our Contributions

This article has its contributions in two folds: First, learning effective word representations based on distributional, syntactic, and relational contexts; and second, employing the learned word representations for the classification of biomedical texts using deep learning-based classification models. It is a major extension of one of our conference papers, [11], by considering larger datasets, more benchmark evaluation datasets, effective application of the learned word representation for text classification using deep learning models, and the comparative evaluation of the classification performance with the vectors learned by one of the existing state-of-the-art methods, GloVe.

#### 1.3.1. Learning Word Representation

This article presents an approach of learning word representation using distributional, syntactic, and relational contexts. The relational contexts take into account how words are in relation to other words. In other words, how a target word is semantically related with context words in a sentence. We say such semantically associated information between the target and context words in a sentence as relational semantic information. The proposed approach incorporates relational semantic information distilled from a large corpus using dependency-based syntactic patterns [10] to augment the distributional representation of words from the same corpus through the neural network-based learning and updating process. We employ dependency-based syntactic patterns to extract long-range and multihop dependencies between a target word, say, *Whipple* and semantically related words such as *arthralgias*, *chronic diarrhea*, *weight loss*, *fever*, and *abdominal pain*, representing symptoms of *Whipple* disease. We extract these semantically related words in the form of semantic triples using the syntactic structures of the dependency tree and further use these triples to augment the distributional representation of the words. The repository of the extracted triples is called the *relational semantic repository*, which is used to augment the distributional information of the words from the given corpus. To start the learning process, we first obtain the initial vectors by singular value decomposition (SVD) of a positive pointwise mutual information (PPMI) matrix produced from the corpus and the relational semantic repository separately. The initial vectors are merged and updated to minimize the loss such that the PPMI value between co-occurring words from the corpus can be correctly predicted. To optimize the least-square minimization objective, we implement a similar objective function as used in the GloVe [4] model. The initial vectors are augmented such that if any of the co-occurring words from the corpus have their word representation in the *relational semantic repository*, we merge the vectors from the corpus and the *relational semantic repository* and jointly optimize them using the gradient descent-based adaptive optimization. As a result, we get enhanced word representations that could be used for various NLP applications.

#### 1.3.2. Biomedical Text Classification

We evaluate the efficacy of the learned word representation using four different neural network-based classification models over two biomedical datasets. Neural network models, in particular, the CNN-based models, have shown exceptional performance in many NLP and text classification tasks compared to traditional ML algorithms. A CNN model performs high-level feature extraction using convolution filters to capture important features during the training process that helps to improve the classification performance. The other neural networks including LSTM have shown remarkable performance for text classification. To evaluate the versatility of the word representation for the classification task, we employ CNN, LSTM, CNN-LSTM, and the bidirectional LSTM (BiLSTM) models.

In brief, the contributions of this article can be summarized as follows.

- It proposes an approach to learn and augment word representation from a corpus using the *relational semantic repository* extracted from the corpus to handle both long- and short-range dependencies among semantically similar words
- It incorporates the strength of pointwise mutual information, singular value decomposition, and neural network-based updation to learn efficient word representations
- It employs the learned word representations to train four deep learning-based classification models, namely, CNN, LSTM, BiLSTM, and CNN-LSTM to classify biomedical texts
- It compares the efficacy of the learned word representations and their classification performance with the word representation learned by one of the state-of-the-art methods, GloVe.

The remaining part of the article is organized as follows.  Section 2 presents a brief review of the existing works on text classification and word representation learning.  Section 3 presents preliminary information about various concepts used in the article.  Section 4 provides detailed description about the proposed approach of learning word representation and biomedical text classification.  Section 5 presents the experimental details, and Section 6 presents theevaluation results. Finally, Section 7 concludes the article and presents future directions of the research.

## 2. Related Works

The text classification problem has been extensively studied in fields such as text analytics, information retrieval, and data mining by means of machine learning techniques in a wide range of applications including text document clustering, sentiment analysis, language identification, and topic labeling [12]. There are different approaches for text classification, and they follow certain processes such as document representation, feature selection or transformation, vector representation, and the application of statistical or machine learning techniques to achieve the desired performance. The popular traditional machine learning (ML) techniques explored by researchers include support vector machine, k-nearest neighbor, naive Bayes, decision tree, and their variants [13, 14]. Biomedical and clinical texts classification has received much attention of researchers using these machine learning techniques [2, 15–17]. However, in the recent years, there has been a drastic shift from traditional ML techniques to modern neural network-based ML classification techniques because of their potential for adaptive learning and generalized prediction. To this end, deep learning models have been widely used in fields such as computer vision, image analysis, and natural language processing, and they have shown outstanding performance in many biomedical applications because of their ability to model the nonlinear and complex patterns and relationships present within the data [18–21]. The deep learning methods use several layers to extract important features from the raw inputs through various learning and transformations at different layers. Raw inputs to deep learning models are presented as their vector representations whose quality affects the performance of NLP tasks such as text classification. The initial vectors are nowadays taken as distributional representation of words in an embedding space which has shown remarkable performance with the deep learning models.

In the recent years, there has been a growing interest in learning distributional word representation from large unstructured corpora [3, 4]. The advancement of various word representation learning techniques to learn a low-dimensional dense representation of words as vectors, commonly known as word embedding, has efficiently solved many NLP problems such as named entity recognition [22], sentiment analysis [23], and sentence classification [24]. In this direction, two renowned neural network-based learning models commonly known as continuous bag of words (CBOWs) and skip-gram (SG) models [25], have been widely used to learn a distributional representation of words. These models exploit the neighboring context words that co-occur on either side of a target word within a fixed context window. CBOW uses surrounding context words to predict a target word while SG uses a current word to predict the surrounding context words. Likewise, GloVe [4] is another familiar model based on the global co-occurrence matrix that minimizes least square loss while predicting global co-occurrence between the target and context words using initial random vectors of desired dimensions. These models learn distributional word representations from the corpus without incorporating any external knowledge. To enhance the quality of word representations and to incorporate some domain knowledge, several studies [7, 26–29] have used external KBs. Yu and Dredze [26] proposed a joint objective of the relation constraint model and CBOW to learn word representation from a corpus and a similarity lexicon (synonymy) by assigning high probabilities to words that appear in the similarity lexicon. Likewise, Xu et al. [27] use the SG training objective function with additional regularization parameters to incorporate relational and categorical information to learn better word representation. In [30], Ghosh et al. applied the vocabulary-driven skip-gram with negative sampling (SGNS) model to learn word representations that are exclusively associated with diseases from a health-related news corpus by incorporating domain knowledge as a vocabulary of terms associated with diseases, symptoms, and their transmission methods. Most of these approaches use either CBOW or SG and its variants like SGNS to jointly optimize them with the linear combination of some additional objective function or some regularizers. Contrary to this, Alsuhaibani et al. [7], in their joint embedding learning, used a linear combination of GloVe and KB-based objective functions to incorporate relations such as synonymy, antonymy, hypernymy, and meronymy from WordNet. All the discussed and other existing approaches use the third-party knowledge base to enhance distributional word representations without extracting entities and their associations directly from the corpus, and hence ignore the relational semantics between words outside of the range of the context window. Furthermore, these models use linear window-based bag-of-word contexts to capture the contextual features from the corpus. Besides this, there is another approach of learning word representation that uses the syntactic contexts produced by the dependency parse tree generated by the parser rather than window-based contexts. To this end, Levy and Goldberg [9] have used dependency-based syntactic contexts and shown that dependency-based embeddings exhibit better functional similarity than the original SG embeddings. Likewise, Komninos and Manandhar [31] have also shown that the dependency-based word embeddings capture better functional properties and improved classification performance. Moreover, recent advancements in NLP have led to a focus on domain-specific tasks by fine-tuning the sizeable pretrained neural language models such as bidirectional encoder representations from transformers (BERTs) [32] for NLP tasks such as named-entity recognition and question answering. Researchers have demonstrated the adaptability of Word2Vec and BERT in the field of biomedical domain to develop models such as BioWordVec [33] and BioBERT [34], as well as other domain-specific models such as SciBERT [35] trained on various scientific and biomedical corpuses, ClinicalBERT [36] trained on clinical notes for various NLP tasks, and MatSciBERT [37] trained on material science publications. Deep learning models that take such trained word representations as input have been employed by researchers to classify unstructured texts documents [38], medical notes [39], health-related social media texts [40], and biomedical text mining tasks [41]. Besides these, handwritten script recognition [42], detection of diseases [43–45], and healthcare solutions [46] involve the potential application of deep learning models.

Word representations learned through the aforementioned algorithms are being used and accordingly evaluated for various NLP applications as they capture contextual features of words. These semantically rich word representation or word vectors are fed as the input to neural networks like CNN and LSTM for performing tasks such as sentiment analysis [47–49] and text classification [24, 50]. As the proposed approach has learned word representation related to the biomedical domain, we evaluate the quality of trained word vectors through a text classification task over biomedical datasets.

## 3. Preliminaries

This section describes the background details of the essential concepts used in the proposed approach. Assume that a corpus *𝒞* consists of *n* documents *d*_1_, *d*_2_,…, *d*_*n*_, and *D* is the collection of target and context words pairs (*w*, *c*) extracted from *𝒞* such that for any target word *w*_*i*_, the context words are the neighboring words *w*_*i*−*ℓ*_,…, *w*_*i*−1_, *w*_*i*+1_,…, *w*_*i*+*ℓ*_ of *w*_*i*_ within a fixed context window *ℓ*. Additionally, *V*_*w*_ and *V*_*c*_ represent the word and context vocabularies of *D*, respectively. Throughout the article, bold letters represent vectors.  Table 1 presents a list of notations and their brief descriptions used in this article.

### 3.1. GloVe

GloVe (https://nlp.stanford.edu/projects/glove/) is a neural network-based method to learn the distributional representation of words in an embedding space, exploiting the global statistical information of words from a text corpus in an unsupervised manner. Given a fixed context window, the algorithm first creates a co-occurrence matrix *M* from the corpus considering the context words (columns of *M*) within a fixed window surrounding a target word (rows of *M*) and then uses the matrix *M* to obtain efficient word representation through the neural network-based learning and updating process. Matrix entries *M*_*i*,*j*_ represent the sum of the reciprocal distances of the co-occurring context words from the target word. The algorithm minimizes the weighted least-square regression loss *J*_*g*_, as shown in equation (1), where *f*(*M*_*w*,*c*_) represents the weight function defined in equation (2) to assign weights between the target word *w* and the context word *c*, and *b*_*w*_ and *b*_*c*_ represent their corresponding bias terms [4]. The hyperparameter *α* and *x*_max_ in equation (2) are assigned 0.75 and 100 values, respectively, to control the overweighting of rare and frequent co-occurrences [4].

(1) $$\begin{array}{c} J_{g}=\frac{1}{2}\underset{w\in V_{w}}{\sum }\underset{c\in V_{c}}{\sum }f\left(M_{w,c}\right){\left(w^{T}\cdot c+b_{w}+b_{c}-\log\left(M_{i,j}\right)\right)}^{2}\text{,} \end{array}$$

(2) $$\begin{array}{c} f\left(M_{w,c}\right)=\min\left\{{\left(\frac{M_{w,c}}{x_{\max}}\right)}^{\alpha },1\right\}\text{.} \end{array}$$

The GloVe algorithm starts the learning process from the randomly initialized vectors of desired dimensions for the target and context words and gradually updates the initial vectors using the stochastic gradient descent (SGD) algorithm. The primary goal of the GloVe algorithm is to minimize the weighted least-square loss such that the word co-occurrence probabilities can be accurately predicted by the dot product of the target and context word vectors.

### 3.2. Pointwise Mutual Information

Word and context associations are mostly represented as the co-occurrence of word and context pair (*w*, *c*) from the corpus. However, a mere co-occurrence count does not include any contextual information; hence, it may not be the best measure of association. Pointwise mutual information (PMI) is another powerful measure of association that quantifies how many times two events (words *w* and *c*) appear together compared with what one might expect if they occurred independently, as defined by equation (3) [51]. Alternatively, the PMI value between the target word *w* and the context word *c* is the log ratio of the joint probability words pair (*w*, *c*) and the product of their marginal probabilities. It gives an estimate of the strength of the association between the target and context words. In the case, when *w* ∈ *V*_*w*_ and *c* ∈ *V*_*c*_ do not co-occur within the fixed window *ℓ* in the corpus, we have*n*_(*w*, *c*)_=0 which causes *PMI*(*w*, *c*)=log(0)=−*∞*. Furthermore, negative PMI values tend to be unreliable unless we have massive corpora. To circumvent these situations, another familiar measure called positive PMI (PPMI) is used which maps negative PMI values to zero using equation (4). It has been shown in [52] that PPMI is a better metric than PMI to obtain the semantic similarity between two words. Equation (4) selects the max of *PMI*(*w*, *c*) and 0 to calculate the PPMI value, as it is preferable to have word pairings with more evidence supporting their similarity a higher score when measuring the word similarity. However, PPMI matrices are highly sparse and require extensive computational resources. One way is to map such sparse matrices into low-dimensional dense vectors for generalization and computational efficiency by employing matrix factorization techniques like SVD.

(3) $$\begin{array}{c} PMI\left(w,c\right)=\log\left(\frac{P\left(w,c\right)}{P\left(w\right)\times P\left(c\right)}\right) \end{array}$$

(4) $$\begin{array}{c} PPMI\left(w,c\right)=\max\;\left\{PMI\left(w,c\right),0\right\}\text{.} \end{array}$$

### 3.3. Singular Value Decomposition

Singular value decomposition (SVD) is a dimensionality reduction technique that factorizes a symmetric matrix *M*_*m*×*n*_ into three matrices *U*, Σ, and *V* in such a manner that *M*=*U*∙Σ∙*V*, where *U* and *V* represent the orthogonal matrices and Σ represents a diagonal matrix of positive real values called singular values. It reduces data dimensions by preserving the main relationship of interest into a low-dimensional representative matrix. To produce *d*dimensional dense vectors, we can decompose matrix *M* into *U*_*m*×*d*_, Σ_*d*×*d*_, and *V*_*d*×*n*_ corresponding to top *d*singular values. In NLP applications, we can produce *d*-dimensional dense matrix $W=U∙\sqrt{\Sigma }$ which is an approximate representative of high dimensional sparse matrix *M* [53]. Furthermore, in word and context situations, we can get the target and context word representative matrices $W=U∙\sqrt{\Sigma }$ and $C=V^{T}∙\sqrt{\Sigma }$ respectively, by decomposing *M* as stated in [53]. These initial representative matrices (*W* and *C*) should satisfy the criteria of minimizing the matrix decomposition error.

## 4. Proposed Approach

This section presents a detailed description of the proposed approach of learning augmented word representation from a large corpus and a relational semantic repository and their application for biomedical text classification.  Figure 2 demonstrates the work-flow of the proposed approach, which comprises methods to produce initial word representation, augment and update the initial word vectors through the relational semantics, and use learned word representation for text classification. It depicts a document crawler to crawl PubMed documents using a set of query patterns. The crawled documents constitute a corpus *C*, which we use to evaluate the proposed approach. The same corpus is exploited to extract the relational semantic information as discussed in [10, 54] and utilized to construct a *relational semantic repository*, *R*_*l*_. The corpus and the *relational semantic repository* are employed to generate the initial word representation by applying SVD on their underlying PPMI matrices.

A detailed description of various processes involved in learning word representation is presented in the following subsections.

### 4.1. Initial Vector Representation

The first step involved in our proposed approach is to initialize vectors of desired dimensions for each target and context words. We augment and update these initial vectors using the *relational semantic repository* and a weighted least-square loss minimization function to obtain enriched embedding. Traditionally, distributed word representations relied on count-based vectors such as tf-idf or SVD based vectors. However, neural network-based word representations that considers the target word and its context within a fixed window have proven to be very effective in various NLP applications. The word representations learned using GloVe [4] and Word2Vec [3] methods have shown their applicability in various NLP applications. However, Levy et al. [53, 55] have shown that neural network-based word representation is analogous in performance to traditional word representation generated by the decomposition of the PPMI matrix formed from the co-occurrence matrix of a corpus. Hence, to include the strength of traditional decomposition-based vectors, the proposed word representation approach adopts the PPMI approach to generate initial word representation by factorizing PPMI matrix using SVD. Accordingly, we first build a co-occurrence *M* using the co-occurrence count of target and context words pairs (*w*, *c*) from corpus *D* with *w* ∈ *V*_*w*_ and *c* ∈ *V*_*c*_. The matrix *M* is then mapped to a PPMI matrix *M*_*p*_, which is further decomposed using SVD to produce *U*, Σ and *V*. Consequently, we obtain initial word representations for the target and context words as matrix *W* and *C* by considering $W=U∙\sqrt{\Sigma }$ and $C=V∙\sqrt{\Sigma }$, respectively. Likewise, we also obtain the initial word representations from the relational semantic repository *R*_*l*_ and represent them as $\hat{W}=U∙\sqrt{\Sigma }$ and $\hat{C}=V^{T}∙\sqrt{\Sigma }$, respectively, for the target and context words. Furthermore, to have better word representation, the resulting initial word representations from the corpus needs to fulfill minimization of the error in matrix decomposition. To minimize error and to incorporate relational semantic information from *R*_*l*_, we augment and update the initial word representation from the corpus in such a manner that the weighted least-square loss is minimum. The augmentation and updating process of the initial word representation is described in the following subsection.

### 4.2. Objective Function Augmentation

In the proposed approach, we adopt the GloVe approach for minimizing the decomposition error to optimize the initial word representation. GloVe learns a low-dimensional dense representation of word vectors from a corpus without incorporating any additional or external relational knowledge. We have discussed its important limitation in Section 1. To address these limitations, we incorporated information from a relational repository into the initial word representation from the corpus by merging the initial word representations from the *relational semantic repository* with the initial word representations from the corpus. We perform this merging of vectors during the optimization process to produce augmented and enhanced word representation. To this end, we define an objective function *J*_*a*_ analogous to the GloVe objective function as shown in equation (5), where *f*(*p*_*w*,*c*_) is a function to assign weight to a co-occurrence pair (*w*, *c*) using equation (6), *p*_*w*,*c*_ is the PPMI value of the pair (*w*, *c*), and *b*_*w*_ and *b*_*c*_ are biases of vectors *w* and *c*, respectively. The vectors *w* and *c* are merged initial word and context vectors of *C* and *R*_*l*_. The merging process of initial vectors is described in the following paragraph.

(5) $$\begin{array}{c} J_{a}=\frac{1}{2}\underset{w\in V_{w}}{\sum }\underset{c\in V_{c}}{\sum }{f\left(p_{w,c}\right)\left({w^{\prime }}^{T}\cdot c^{\prime }+b_{w}+b_{c}-\log\left(p_{w,c}\right)\right)}^{2}\text{,} \end{array}$$

(6) $$\begin{array}{c} f\left(p_{w,c}\right)=\min\left\{{\left(\frac{p_{w,c}}{\max_{\forall w,c\in D}\left(p_{w,c}\right)}\right)}^{\alpha },1\right\}\text{.} \end{array}$$

We consider three categories of words from the vocabulary *V* of the (*w*, *c*) pair collection *D* based on their presence or absence in the vocabulary, *𝒱*, of *R*_*l*_. These include *D*_∧_, *D*_∼_, and *D*_⊕_, which are described in the following paragraphs.

- *D*_∧_={(*w*, *c*)|*w* ∈ *𝒱*, *c* ∈ *𝒱* and(*w*, *c*) ∈ *D*} it represents the category of (*w*, *c*) pairs in which both the target and context words are the members of *𝒱*.
- *D*_∼_={(*w*, *c*)|*w* ∉ *𝒱*, *c* ∉ *𝒱* and(*w*, *c*) ∈ *D*} it represents the category of (*w*, *c*) pairs wherein neither the target nor the context word is a member of *𝒱*.
- *D*_⊕_={(*w*, *c*)|*w* ∈ *𝒱*, *c* ∉ *𝒱*∨(*w* ∉ *𝒱*, *c* ∈ *𝒱* and(*w*, *c*) ∈ *D*)} it represents the category of (*w*, *c*) pairs in which either the target or the context word is a member of *𝒱*.

Each of the three categories of word pairs requires to be handled accurately while merging the initial vectors of *R*_*l*_ and *C*. Consider the first case *D*_∧_ wherein both the target and context words are the member of *𝒱*, we have initial vectors from *R*_*l*_ as well as *C* for the target and context words *w* and *c*. These initial vectors are merged in such a way that the resultant vector corresponding to the target word *w* is $w^{\prime }=0.5*\left(w+\hat{w}\right)$ and the resultant vector corresponding to the context word *c* is $c^{\prime }=0.5*\left(c+\hat{c}\right)$. It should be noted that **w** and **c** are vectors from , while $\hat{w}$ and $\hat{c}$ are vectors from *R*_*l*_.

Likewise, in the second case, *D*_∼_={*w*, *c* wherein neither the target word nor the context word is a member of *𝒱*, we have the initial vector representation of words *w* and *c* from the corpus only. In this case, as *w* and *c* are not found in *R*_*l*_, no merging is needed. As a result, the resultant vector corresponding to *w* and *c* are equal to **w** and **c**, respectively, i.e., **w**′=**w** and **c**′=**c**. Similarly, for the third case **D**_⊕_ wherein either the target or the context word is contained in *𝒱*, we have any of the two word's (target or context) initial vector representation in both *C* and *R*_*l*_. In this case, either we use the target or the context word's merged initial vector representation depending upon which word belongs to both the repository. If we have the target word in both the repository, the resultant target word is $w^{\prime }=0.5*\left(w+\hat{w}\right)$, and if we have the context word from both the repository, then the resultant context word is $c^{\prime }=0.5*\left(c+\hat{c}\right)$.

### 4.3. Adaptive Updation of Parameters

Gradient descent techniques are widely used optimization techniques for parameter updation during the training of neural networks. Just like the GloVe model, we use the Adagrad [56] gradient descent technique to update parameters during the learning process. Adagrad is an adaptive update algorithm, which automatically adjusts the learning rate. The gradient for the target and context words and their corresponding biases are calculated using the following equations:

(7) $$\begin{array}{c} \frac{\delta J}{\delta w^{\prime }}=g_{t,w^{\prime }}\\ =\underset{c\in V_{c}}{\sum }f\left(p_{w,c}\right)\left({w^{\prime }}^{T}\cdot c^{\prime }+b_{w}+b_{c}-\log\left(p_{w,c}\right)\right)∙c^{\prime }\text{,}\\ \frac{\delta J}{\delta c^{\prime }}=g_{t,c^{\prime }}\\ =\underset{w\in V_{w}}{\sum }f\left(p_{w,c}\right)\left({w^{\prime }}^{T}\cdot c^{\prime }+b_{w}+b_{c}-\log\left(p_{w,c}\right)\right)∙w^{\prime }\text{,}\\ \frac{\delta J}{\delta b_{w}}=g_{t,b_{w}}\\ =\underset{c\in V_{c}}{\sum }f\left(p_{w,c}\right)\left({w^{\prime }}^{T}\cdot c^{\prime }+b_{w}+b_{c}-\log\left(p_{w,c}\right)\right)\text{,}\\ \frac{\delta J}{\delta b_{c}}=g_{t,b_{c}}\\ =\underset{w\in V_{w}}{\sum }f\left(p_{w,c}\right)\left({w^{\prime }}^{T}\cdot c^{\prime }+b_{w}+b_{c}-\log\left(p_{w,c}\right)\right)\text{.} \end{array}$$

AdaGrad efficiently handles the sparse data by performing larger updates for rarely occurring words while smaller updates for frequently occurring words. Equation (8) is used for updating target word vectors,

(8) $$\begin{array}{c} {w^{\prime }}^{t+1}={w^{\prime }}^{t}-\frac{\eta }{\sqrt{\sum_{\tau =1}^{t}g_{\tau ,w^{\prime }}^{2}}}*\left(g_{t,w^{\prime }}\right)\text{,} \end{array}$$

where **w**′ represents a combined target word vector, *g*_*t*,*w*_ represents gradient at time *t*, and *g*_*τ*,*w*_^2^ denotes squared gradient at time *τ* for **w**′. Likewise, equations (9)–(11) are used for updating the merged context word vector and the target and context word biases, respectively.

(9) $$\begin{array}{c} {c^{\prime }}^{t+1}={c^{\prime }}^{t}-\frac{\eta }{\sqrt{\sum_{\tau =1}^{t}g_{\tau ,c^{\prime }}^{2}}}*\left(g_{t,c^{\prime }}\right)\text{,} \end{array}$$

(10) $$\begin{array}{c} b_{w}^{t+1}=b_{w}^{t}-\frac{\eta }{\sqrt{\sum_{\tau =1}^{t}g_{\tau ,b_{w}}^{2}}}*\left(g_{t,b_{w}}\right)\text{,} \end{array}$$

(11) $$\begin{array}{c} b_{c}^{t+1}=b_{c}^{t}-\frac{\eta }{\sqrt{\sum_{\tau =1}^{t}g_{\tau ,b_{c}}^{2}}}*\left(g_{t,b_{c}}\right)\text{.} \end{array}$$

### 4.4. Deep Learning Models

This section presents a detailed description of deep learning models used for the text classification. The deep learning models, along with the word embeddings as the input, are proving to be very effective for text classification. These are essentially machine learning models with better intelligence, efficient learning ability, high accuracy, and robust performance. The most popular basic deep learning models used for text classification are CNN and LSTM networks and their variants such as BiLST and CNN-LSTM. All these models take a sequence of input vectors corresponding to the textual data and exploit these vectors to capture important features helpful to map the text into their respective labels. The texts to be classified are first preprocessed by tokenizing and removing symbols, punctuation marks, numbers, and stopwords. The pre-processed text documents consisting of *k* tokens are then transformed into a sequence of *n*-dimensional vectors, where vectors correspond to learned word representations obtained either by the proposed approach or other state-of-the-art-approaches like GloVe. All the deep learning models used for the text classification task are given the input text document as a sequence of *n*-dimensional *k* vectors forming a *k* × *n* embedding matrix corresponding to *k* tokens. Given the pre-processed text document *T* with *k* tokens and *x*_1_, *x*_2_,…, *x*_*k*_ vectors corresponding to *k* tokens, the embedding matrix can be represented by (12), where ⊕ represents the concatenation operation over the vectors.

(12) $$\begin{array}{c} T=x_{1}⊕x_{2}⊕\ldots ⊕x_{k}\text{.} \end{array}$$

We consider *k* of fixed length (*k* = 25) to form the embedding matrix. The embedding matrices thus formed constitute an embedding layer for each model, and these embedding matrices are then fed into the different deep learning models for learning high-level features to perform efficient classification. The deep learning models used in this article for biomedical text classification are discussed in the following sub-sections.

#### 4.4.1. Convolutional Neural Network (CNN)

A CNN model comprises various layers for converting texts into embedding matrix and learning high-level features bypassing the embedding matrix through the convolution layer and the intermediate outputs through the max-pooling layer and fully connected dense layers to predict the class labels. The given text is preprocessed by tokenizing and removing symbols, punctuation, number, and stopwords. The preprocessed tokens, say *k* tokens per text document, are then mapped into an embedding matrix (a sequence of *k* vectors) at the embedding layer using the learned word representation. The embedding matrices formed from the input texts are feed as input to the convolution layer, which employs filters of different width by convolving them through the embedding matrices to extract high-level features and accordingly creates feature maps. A filter, say, *ℱ* ∈ *ℝ*^*m*×*n*^ of width *m* convolves through the embedding matrix *T* with stride *s* to create the feature map *c*_*i*_ determined by (13), where *∗* is the convolution operation, *T*_*i*:*i*+*m*−1_ represents the vectors from *w*_*i*_ to *w*_*i*+*m*−1_ of *T* convolved by filter *ℱ*, *b*_*i*_ is the biased term, and *f* denotes an activation function. An activation function *rectified linear unit*(ReLU) is used to introduce nonlinearity to the system that can be represented by equation (14).

(13) $$\begin{array}{c} c_{i}=f\left(F*T_{i:i+m-1}+b_{i}\right)\text{,} \end{array}$$

(14) $$\begin{array}{c} f\left(x\right)=\max\;\left\{0,x\right\}\text{.} \end{array}$$

The feature maps are further passed through a max-pooling layer, which selects the max-value from the feature maps corresponding to each filter *ℱ* to form a max-pooled feature vector. To control overfitting problems, drop out is used that drops some neurons while keeping the others with some probability. The last layer of the network is the fully connected dense layer, which predicts the class probabilities using the *softmax* activation function [57]. The detailed description of the basic CNN architecture applied in our experiment can be found in [50]. The categorical cross-entropy loss function is used to calculate the loss while the AdaDelta [58] algorithm is used to update and optimize the parameters.

#### 4.4.2. Long Short-Term Memory (LSTM)

LSTM networks are a slightly tweaked form of recurrent neural networks (RNN) to make them suitable for text classification tasks. LSTM networks contain “memory cells,” which are controlled by input, output, and forget gates. The gates control the inflow and outflow of information through the memory cells. The input gate adds new information to the cell and uses an activation function to regulate the value to be added. Similarly, the forget gate discards some information from the current content of the memory cell, while the output gate decides how much information should be forwarded to the next hidden state. LSTM uses two-way storage of information where short-term recent history is stored as activation of neurons while the long-term memory stores weight, which gets modified based on the backpropagation. During forward pass, the input and output gates learn when to allow the activation to get into the internal state and when to pass it to the output state, respectively. When these entry and exit points are closed, the activation is captured inside the memory cell and hence does not expand, shrink, or affect the output of any intermediate state across multiple time steps. Similarly, during backpropagation, the gradients neither vanish nor explode across time steps. This allows LSTM to capture long-term dependency effectively in comparison to simple RNN.

As stated above, the memory cells consist of input, output, forget gates, and a candidate memory cell, and their values are updated at a time-step *t* for the input vector *w*_*t*_ using the following equations:

(15) $$\begin{array}{c} i_{t}=\sigma \left(W_{i}.\left[h_{t-1};w_{t}\right]+b_{i}\right)\text{,}\\ f_{t}=\sigma \left(W_{f}.\left[h_{t-1};w_{t}\right]+b_{f}\right)\text{,}\\ o_{t}=\sigma \left(W_{o}.\left[h_{t-1};w_{t}\right]+b_{o}\right)\text{,}\\ g_{t}=\tanh\;\left(W_{r}.\left[h_{t-1};w_{t}\right]+b_{r}\right)\text{,}\\ c_{t}=i_{t}⊙g_{t}+f_{t}⊙c_{t-1}\text{,}\\ h_{t}=o_{t}⊙\tanh\left(c_{t}\right)\text{,} \end{array}$$

where ⊙ represents elementwise multiplication, *σ* represents the sigmoid function, and *W*_*i*_, *b*_*i*_, *W*_*f*_, *b*_*f*_, *W*_*o*_, and *b*_*o*_ represent input, forget, and output gates' parameters. The final hidden vector obtained from the LSTM cell representing high-level features for the input texts is fed into a dense layer with the softmax activation function, which maps the output into the probabilities of classifying the texts into their corresponding class labels. Softmax activation function is frequently employed to solve multiclass classification problems. It computes the relative probabilities of high data points (vector obtained from the LSTM cell representing high-level features), indicating that the data points belong to a particular class. We have applied the LSTM model for biomedical text classification tasks in the experimental section.

#### 4.4.3. Bidirectional Long Short-Term Memory (BiLSTM)

Bidirectional LSTM (BiLSTM) is an extension to the unidirectional LSTM to incorporate both the historical and future contexts by introducing another hidden layer. BiLSTM captures the contextual information from both ways, reading the inputs in both the forward (normal way) and reverse directions, which is quite advantageous in text classification tasks. If the hidden state for the forward sequence context is represented by $\overset{⟶}{h}$ and the backward sequence context is represented by $\overset{⃖}{h}$, then the output of the *i*^*th*^ word is given by the following equation:

(16) $$\begin{array}{c} h_{i}=\left[\overset{⟶}{h}⊕\overset{⟵}{h}\right]\text{,} \end{array}$$

where ⊕ represents elementwise sum of vectors $\overset{⟶}{h}$ and $\overset{⟵}{h}$. The *softmax* function is used to map the text into the corresponding label.

#### 4.4.4. CNN-LSTM

The CNN-LSTM model consists of the CNN layer to extract the local *n*-gram features from the input data for the LSTM layer, which interprets the features for sequence prediction across time steps. We can say that the CNN-LSTM model comprises two submodels, CNN and LSTM. For the text classification task, the CNN submodel comprises a 1*D* convolutions layer followed by a 1*D* max-pooling layer to capture and consolidate important high-level features as vectors. The max-pooled feature vectors are then fed into the LSTM layer, which captures the long-distance dependency features and gives the final text representation. It is further passed through a dense layer with the *softmax* activation function to map the text into corresponding class probabilities.

## 5. Experimental Setup and Results

We use a biomedical text corpus for learning word representation and evaluate the learned word vectors over multiple benchmark datasets for two evaluation tasks: *word similarity* and *concept categorization*. We also present an application of the learned word representation for the biomedical text classification task. The following subsections briefly describe the corpus and the *relational semantic repository* used for experimentation, the experimental setup, and the evaluation results over various benchmark datasets.

### 5.1. Corpus and the Relational Semantic Repository

The proposed approach is evaluated over a biomedical text corpus crawled from PubMed (https://www.ncbi.nlm.nih.gov/pubmed/) database, which is an online repository of thousands of abstracts and citations related to various biomedical fields such as health, biomedicine, bioengineering, and life and behavioural sciences. These biomedical abstracts encapsulate many disease-related useful information such as disease names, their associated symptoms, vectors, pathogens, etiologies, transmitting agents, and drug-related information. PubMed gives access to the abstracts of biomedical literature through its NCBI Entrez systems API (*axis 2.1.6.2* (https://axis.apache.org/axis2/java/core/)) by querying its server using desired keywords. We retrieved 67516 abstracts, called corpus *C*, related to cholera, dengue, diarrhoea, influenza, leishmaniasis, malaria, and meningitis diseases by querying the PubMed database. The document retrieval process is discussed in detail in [10, 54]. Moreover, we created the *relational semantic repositoryR*_*l*_ from the relation triples (<entity_*i*_, relation, entity_*j*_>) extracted from the corpus. *R*_*l*_ consists of disease symptom and their associations in the form of semantic triples, which are extracted using typed dependencies generated by Stanford parser (https://nlp.stanford.edu/software/lex-parser.shtm) and filtered by employing MetaMap (https://metamap.nlm.nih.gov/). The process of extraction of relation triples is discussed in [10, 54].

### 5.2. Experimental Setup

The documents from the corpus *C* are tokenized and preprocessed by eliminating punctuation marks, stopwords, and numbers. We first generate a co-occurrence matrix from the corpus using the co-occurrence count of the target and context words within the fixed context window. The experimental evaluation is performed on two different context window sizes *ℓ* ∈ {5,10} to consider the neighboring context of a target word. For example, for *ℓ* = 5, the context words for a target word are 5 prior and 5 following words to the target within the document. The co-occurrence matrix thus formed is converted into the PPMI matrix according to the method discussed in Section 4. The PPMI matrix is further factorized using SVD to obtain the initial vector representation of corpus words. The same procedure is applied to obtain initial word representation from *R*_*l*_. We consider two different dimensions *d* ∈ {100,200} of the initial vectors to report the evaluation results of the proposed approach. To optimize the initial vectors by minimizing the least-square loss, we used the objective function defined in equation (5). We used AdaGrad [56], which is an SGD-based adaptive update algorithm for updating of parameters and optimizing the vectors. The initial learning rate, *η*, is adjusted to 0.05 for updating parameters. The algorithm of the proposed approach was executed for 50 iterations to converge it into an optimal solution. Consequently, we received two sets of improved vectors, one for the target words called WE and the other for the context words called CE. Furthermore, their combined vectors, namelyMerged are considered by taking the average of the corresponding target and context vectors for a particular word from the vocabulary *V*_*w*_. We considered Merged vectors because the authors in [4] reported that the merged vectors perform better than either of the word and context vectors. We have reported the evaluation results of all the three forms (target word, context word, and the merged form) of the vectors learned by the proposed approach and the corresponding form of the vectors (GloVe_W, GloVe_C, and GloVe_Merged) learned by GloVe.

#### 5.2.1. Parameters Setting for Biomedical Text Classification Models

For the biomedical text classification task, we employed four basic neural network-based models: CNN, LSTM, BiLSTM, and CNN-LSTM, as discussed in Section 4 considering various parameter settings for the underlying models. We executed each model for 100 epochs and report the best results for each model in terms of training and validation accuracy. For all the models, we used Ada de lta optimizer [58], which dynamically adapts over time and does not require hyperparameter tuning. Furthermore, we used the *categorical cross entropy* loss function to estimate the loss of a model for updating weights. For the CNN model, the initial filter and softmax weights are sampled from the interval [−0.1, 0.1]. We applied 100 filters of width m = 3 and stride s = 1, max-pooling of size 2, a dropout of 0.5 prior to the dense layer, and *ℓ*_2_ regularization of 0.03 at the convolution layer. Similarly, for the LSTM model, we used 256 hidden units of LSTM, and for the remaining two models, the parameters settings remain the same.

We evaluate the quality of vectors learned through the proposed approach in terms of two assessment tasks that include *word similarity* and *concept categorization*. We also provide an application of the learned word representation to classify biomedical texts into different labels using four neural network-based classification models.

#### 5.2.2. Word Similarity

For word similarity evaluation, we compare the cosine similarity of word pairs determined using the learned word representation against the similarity scores assigned by the human annotator to the corresponding word pairs. The evaluation is based on the principle that the semantics of words are preserved by the trained word representation if we have positive correlations between the calculated similarity value and the human-rated similarity value for the word pairs. In this regard, we use Spearman's rank correlation coefficient to find the correlation between the calculated similarity value and the annotated similarity value for the word pairs of the benchmark datasets. The quality of word vectors learned using the proposed approach is evaluated over fifteen benchmark datasets: *BioSimLex* [59], *BioSimVerb* [59], *MEN* (https://clic.cimec.unitn.it/elia.bruni/MEN.html), *MTurk* [60], *RG65* [61], *RW* (https://www-nlp.stanford.edu/%20lmthang/morphoNLM/) [62], *SCWS* [63], *SimLex999* [64], *TR9856* [65], *UMNSRS-Rel* [66], *UMNSRS-Sim* [66], *VERB143* [67], *WS353* [68], *WS353R* [68], and *WS353S* [68]. *BioSimLex* and *BioSimVerb* datasets cover the concept pairs in biomedicine and comprise 988 noun pairs and 1000 verb pairs, respectively [59]. *MEN*, *MTurk*, and *RG65* datasets contain collection of 3000, 771, and 66 English word pairs, respectively, for evaluation of semantic similarity and relatedness. *RW* is a rare word dataset containing 2034 low-frequency word pairs to check the rare word representation [62], while *SCWS* contains 2003 word pairs along with their contexts [63]. Similarly, *SimLex999* contains different POS-category word pairs together with the correctness level and association strength [64]. Likewise, the *UMNSRS-Sim* and *UMNSRS-Rel* datasets contain 566 and 587 pairs of medical terms, respectively, for evaluation of semantic similarity and relatedness [66, 69]. The *VERB143* dataset contains 143 annotated verb pairs for similarity task. Similarly, *WS353* is the original data and its two subsets *WS353S* and *WS353R*, containing 353, 203, and 252 word pairs, respectively, associated with semantic similarity and relatedness [68].

We compare the performance of word representations learned using the proposed approach and the GloVe method for the word similarity task. We have considered different window sizes *ℓ* ∈ {5,10} and vector dimensions *d* ∈ {100,200} to assess the window size and dimension effects on the learned vectors. The *word similarity* evaluation results on various combinations of vector dimension and window size are presented in Tables 2–5. It can be observed from these tables that the word vectors trained using the proposed approach report the best results for all combinations of the window size and vector dimension compared to the GloVe-based vectors except for four instances over the *RW*, *VERB143*, and *WS353* datasets. Although in these four instances (two in the case of *RW* and one each in the case of *VERB143* and *WS353*), GloVe-based vectors report better results, and the difference in the performance between the trained vectors using the proposed approach and GloVe is not significant. Another interesting observation is that at *ℓ*=10, the word vectors using the proposed approach perform better on all the datasets for both dimensions *d*=100 and 200. It signifies that long-range dependencies are also vital. The best performance in the case of each dataset over different combinations of the window size and vector dimension is highlighted in bold typeface. Furthermore, we can also observe from these tables that word vectors learned using the proposed approach perform significantly better over *UMNSRS-Rel* and *UMNSRS-Sim* datasets in comparison to the GloVe-based vectors. The results from these tables also show that *CE* and *Merged* vectors learned using the proposed approach dominate over all other vectors. Similarly, the other interesting insights may be inferred from these tables.

#### 5.2.3. Concept Categorization

It is another way of evaluating the quality of word representations wherein the set of concepts is grouped into distinct categories. It is based on the clustering of vectors into distinct groups, and the performance is measured by the number of concepts each cluster has from a given category. Here, the *purity* metric is used, wherein 100% purity specifies that the given category is completely reproduced and hence vectors are of highest quality, whereas 0% purity specifies that the cluster quality is worst. We used seven benchmark datasets: *AP* [70], *BLESS* [71], *Battig* [72], *ESSLI_1a* (https://wordspace.collocations.de/doku.php/data:esslli2008:concrete_nouns_categorization), *ESSLI_2b* (https://wordspace.collocations.de/doku.php/data:esslli2008:abstract_concrete_nouns_discrimination), *ESSLI_2c* (https://wordspace.collocations.de/doku.php/data:esslli2008:verb_categorization), and *Ohta-10-bio-words* (https://github.com/spyysalo/wvlib/tree/master/word-classes/Ohta-10-bio-words) for the evaluation of learned word vectors using the *concept categorization* task. The *AP* dataset contains 402 words with 21 concept categories [70], *BLESS* contains 200 concepts with 17 semantics classes [71], *Battig* contains 5231 words listed in 56 taxonomic categories [72], *ESSLI_1a* contains 44 concrete nouns belonging to 6 semantic categories, *ESSLI_2b* contains 40 nouns classified into three classes, *ESSLI_2c* contains 45 verbs belonging to 9 semantic classes, and *Ohta-10-bio-words* contains 12 word classes of the biomedical domain.

The evaluation results corresponding to the *concept categorization* task on various combinations of vector dimension and window size are presented in Tables 6–9. It can be observed from these tables that the word vectors trained using the proposed approach show the best performance for all combinations of the window size and vector dimension compared to the GloVe-based vectors except for the five instances over *ESSLI_2a*, *ESSLI_2b*, and *ESSLI_2c* datasets. Among these five instances, the GloVe-based vectors show best performance in three cases over the *ESSLI_2c* dataset and one case each over *ESSLI_2a* and *ESSLI_2b* datasets. The best performance in the case of each dataset in these tables is highlighted in bold typeface. Furthermore, it can be observed from these tables that for each of the four combinations of the window size and vector dimension, the vectors learned by both the approaches show the worst performance over the Battig dataset, whereas the best performance switches between *ESSLI_2a* and *ESSLI_2b* datasets. Moreover, the merged vectors using the proposed approach dominate the performance and show the best results in most of the cases.

## 6. Comparative Analysis and Evaluation for Biomedical Text Classification Tasks

We investigate the performance of learned word embeddings on two different text classification tasks: one is binary classification task over the *BioText Berkeley* dataset and the other one is multiclass classification over the *PubMed RCT 20K* dataset. The details of the datasets and text classification performances are presented in the following subsections.

### 6.1. Comparative Analysis on the BioText Berkeley Dataset

The *BioText Berkeley* dataset (https://biotext.berkeley.edu/dis_treat_data.html) is a benchmark dataset containing labeled sentences of 100 titles and 40 abstracts obtained from MEDLINE 2001 and labeled based on the contents of individual sentences [73]. The sentences are labeled based on the roles and relationships of disease and treatment relations considering eight different categories. During dataset preprocessing, we discarded the two categories, namely, “vague” and “to_see.” Thereafter, remaining categories are grouped into two classes, wherein the first class contains all the disease- and treatment-related sentences while the remaining sentences constitute the second class. Finally, the curated dataset is considered as an evaluation dataset for the binary text classification problem. The final dataset contains 3415 labeled sentences.

Following the dataset curation process, the four neural network-based classification models discussed in Section 5 are trained, and underlying results in terms of training and validation accuracy are presented in Tables 10–13. The best results corresponding to the word vectors trained using both the proposed approach and the GloVe method for every combination of the window size and vector dimension are shown in bold typeface. It can be observed from these tables that, in most of the cases, classification accuracy using the vectors trained by the proposed approach is significantly better. An interesting observation from these tables is that CE and WE vectors trained using the proposed approach achieve best performances in most of the cases in terms of training and validation accuracies for various combinations of the window size and vector dimension. Therefore, it can be inferred that averaging CE and WE does not show impressive results in case of the text classification task compared to concept categorization and word similarity tasks where merged vectors have shown good results. Furthermore, among the four neural network-based classification models, the CNN-LSTM model shows the best performance followed by the CNN model. In contrast, the BiLSTM model shows the worst performance.

### 6.2. Comparative Analysis on the PubMed RCT 20K Dataset

The efficacy of the trained word vectors using both the approaches is evaluated over another benchmark dataset *PubMed RCT 20K* [74], which is associated with the biomedical domain. The *PubMed RCT 20K* dataset is extracted and curated from PubMed for sequential sentence classification consisting 20000 abstracts of randomized-controlled trials [74]. Each sentence of the dataset is labeled based on its role in the abstract considering that the sentences can be related to five different categories: *background*, *objective*, *method*, *result*, or *conclusion* [74]. The original dataset was preprocessed to filter the numbers, symbols, and stopwords. As a result, the final dataset comprises 176560 training and 29667 validation sentences. Like the *BioText Berkeley* dataset, we trained the same set of four neural network-based classification models. The underlying results in terms of training and validation accuracies are presented in Tables 14–17. It can be observed from these tables that there is a slight increase in the training and validation accuracies with the increase in the vector dimension and the context window size. Furthermore, in contrast to the *BioText Berkeley* dataset, we can observe from these tables that the BiLSTM and LSTM models perform better than the CNN and CNN-LSTM models. This may be because the dataset is sequential and the sentences are sequentially associated with each other. The CNN model shows the worst performance in comparison to the other models. In this dataset also, *CE* and *WE* vectors show better performance in comparison to the Merged vector. Similarly, the other interesting observations can be inferred from these tables.

## 7. Conclusion and Future Works

Biomedical text classification is becoming important to extract valuable information from the proliferating biomedical repositories, and deep learning has encouraged researchers to develop neural network-based classification models for efficient text classifications using low-dimensional dense vectors (*aka* word embeddings). In this article, we presented a method of incorporating relational semantic information of distant words and the words having infrequent co-occurrence within the corpus in the distributional representation of words through the augmentation of vectors from a corpus of the *relational semantic repository* to learn enriched word representation. The effectiveness of the proposed approach is evaluated by performing *word similarity* and *concept categorization* tasks over various benchmark datasets using the learned word vectors. We have also applied the learned word vectors for classifying biomedical texts and found that they perform significantly better in comparison to the vectors learned by the widely used GloVe model. Since *relation mining* is one of the well-studied problems in the biomedical domain, we have considered the biomedical domain as one of the potential application domains for our proposed word representation method based on the distributional and relational contexts. However, the proposed approach is generic and can be applied to any domain having the required relation triplets. Exploiting external knowledge bases along with the distributional and relational contexts to further improve the word representations is an interesting direction of future research.

## Figures and Tables

**Figure 1:** Dependency relation graph of the example sentence produced by the Stanford NLP parser using the visualization tool *DependenSee 3.7.0*. The image is adopted from one of our previous works [10].

**Figure 2:** Proposed framework for augmented word representation learning and text classification.

**Table 1:** Various notations and their descriptions.

Notations	Descriptions
*w*, *c*	A target word and a context word, respectively
*𝒞*	Corpus containing *n* documents *d*_1_, *d*_2_,…, *d*_*n*_
*D*	Containing the target and context word pairs (*w*, *c*) extracted from *𝒞*
*V*_*w*_, *V*_*c*_	The target and context words vocabularies of the collection *D*, respectively
*n*_(*w*, *c*)_	(*w*, *c*) pairs count in *D*
*n*_*w*_, *n*_*c*_	Counts of *w* and *c*, respectively, in *D* such that $n_{w}=\sum_{\hat{c}\in V_{c}}n_{\left(w,\hat{c}\right)}$ and $n_{c}=\sum_{\hat{w}\in V_{w}}n_{\left(\hat{w},c\right)}$
*M*	Matrix representing association between every pair of target and context words, wherein rows denote target word vectors and columns denote context word vectors
*M*_*i*,*j*_	Matrix entries representing the association between *i*^*th*^ target word *w*_*i*_ ∈ *V*_*w*_ and *j*^*th*^ context word *c*_*j*_ ∈ *V*_*c*_
*R*_*l*_	Relational semantic repository extracted from the corpus *C*
*𝒱*	Vocabulary of *R*_*l*_

**Table 2:** Word similarity performance with *ℓ*=5 and *d*=100.

Word embeddings	BioSimLex	BioSimVerb	MEN	MTurk	RG65	RW	SCWS	SimLex999	TR9856	UMNSRS-rel	UMNSRS-sim	VERB143	WS353	WS353R	WS353S
GloVe_W	0.37086	0.02425	0.08833	0.19136	−0.12219	0.18913	0.32734	0.08983	0.14776	0.02051	0.12093	**0.20339**	0.26537	0.17454	0.28847
GloVe_C	0.37704	0.0234	0.08882	0.19213	−0.11486	0.18979	0.32471	0.08923	0.14850	0.02298	0.12216	0.20214	0.26471	0.17847	0.29069
GloVe_Merged	0.38046	0.01684	0.08901	0.19784	−0.11080	**0.19142**	0.32250	0.08593	0.14683	0.02333	0.12801	0.17483	0.26312	0.17616	0.29588
WE	0.38656	0.09145	0.16012	0.19378	0.08606	0.16619	0.36104	0.15773	0.16101	0.23448	0.33379	0.17740	0.28174	**0.24885**	0.30282
CE	0.3864	0.08932	0.15778	0.19637	0.06870	0.15468	0.36262	**0.16656**	**0.16486**	**0.25085**	0.34071	0.16746	**0.28344**	0.23962	**0.31748**
Merged	**0.41983**	**0.10333**	**0.17876**	**0.22560**	**0.13349**	0.16765	**0.37026**	0.16420	0.15974	0.24083	**0.34355**	0.19662	0.27340	0.24228	0.29602

Bold means the best performance in the case of each dataset.

**Table 3:** Word similarity performance with *ℓ*=5 and *d*=200.

Word embeddings	BioSimLex	BioSimVerb	MEN	MTurk	RG65	RW	SCWS	SimLex999	TR9856	UMNSRS-rel	UMNSRS-sim	VERB143	WS353	WS353R	WS353S
GloVe_W	0.39595	0.02102	0.08633	0.18420	−0.10868	0.19159	0.33133	0.09255	0.14876	0.02863	0.11977	0.20532	**0.27138**	0.1856	0.28586
GloVe_C	0.38942	0.02463	0.08613	0.18368	−0.11569	0.19241	0.33356	0.09008	0.14976	0.02911	0.11795	0.20424	0.27077	0.18893	0.29353
GloVe_Merged	0.39252	0.0167	0.08978	0.18971	−0.1144	**0.19416**	0.32867	0.08579	0.14863	0.03666	0.13204	0.16467	0.26551	0.18294	0.29706
WE	0.45936	0.13931	0.22985	0.34154	**0.16416**	0.17521	0.37285	**0.17074**	0.16225	0.21659	0.31450	0.23520	0.23407	0.18545	0.31335
CE	0.45911	0.14452	0.22756	**0.34159**	0.15423	0.16408	**0.37965**	0.16941	**0.16867**	**0.23040**	**0.31535**	**0.24051**	0.26612	**0.22927**	**0.33163**
Merged	**0.46832**	**0.15000**	**0.23151**	0.33007	0.12302	0.15321	0.37304	0.15882	0.16605	0.22527	0.30895	0.208215	0.22719	0.19314	0.29428

Bold means the best performance in the case of each dataset.

**Table 4:** Word similarity performance with *ℓ*=10 and *d*=100.

Word embeddings	BioSimLex	BioSimVerb	MEN	MTurk	RG65	RW	SCWS	SimLex999	TR9856	UMNSRS-rel	UMNSRS-sim	VERB143	WS353	WS353R	WS353S
GloVe_W	0.41447	0.03500	0.11218	0.25121	−0.08405	0.19361	0.34490	0.10936	0.14681	0.08276	0.16010	0.25775	0.23949	0.15827	0.27814
GloVe_C	0.40711	0.034104	0.11319	0.25104	−0.07161	0.19433	0.34930	0.10657	0.14861	0.08063	0.15738	0.24971	0.24406	0.1695	0.27649
GloVe_Merged	0.42232	0.03079	0.11085	0.24424	−0.07091	0.19534	0.34576	0.10382	0.14725	0.08224	0.16911	0.23834	0.24284	0.16355	0.29231
WE	0.43159	0.13004	0.19873	**0.28795**	0.13609	**0.21529**	**0.37697**	0.15218	0.15606	0.25885	0.33819	0.28255	0.34254	0.27483	0.40136
CE	**0.45262**	0.13312	0.20081	0.28509	0.18909	0.17872	0.37275	**0.15449**	0.15126	0.22989	0.32402	**0.28431**	**0.34823**	**0.31235**	**0.40330**
Merged	0.43254	**0.17497**	**0.21834**	0.27677	**0.22149**	0.13459	0.37611	0.15299	**0.15817**	**0.28289**	**0.35350**	0.18635	0.28867	0.25955	0.32509

Bold means the best performance in the case of each dataset.

**Table 5:** Word similarity performance with *ℓ*=10 and *d*=200.

Word embeddingss	BioSimLex	BioSimVerb	MEN	MTurk	RG65	RW	SCWS	SimLex999	TR9856	UMNSRS-rel	UMNSRS-sim	VERB143	WS353	WS353R	WS353S
GloVe_W	0.43207	0.02696	0.10992	0.25905	−0.08043	0.19756	0.33868	0.10524	0.14693	0.07269	0.14784	0.25767	0.23913	0.15315	0.27493
GloVe_C	0.43398	0.02142	0.11191	0.26266	−0.07475	0.19811	0.3446	0.10384	0.14785	0.08083	0.15536	0.25638	0.23976	0.15199	0.27944
GloVe_M erged	0.44134	0.02201	0.11245	0.25225	−0.07852	0.19850	0.34179	0.09961	0.14727	0.08368	0.16740	0.23064	0.23776	0.15446	0.28936
WE	**0.47840**	0.13275	0.20673	0.25842	0.18457	0.17788	0.38499	0.16691	0.15209	0.22026	0.32647	0.29077	**0.34063**	**0.28352**	**0.40837**
CE	0.46382	0.13086	0.20928	0.26134	0.16582	**0.21132**	**0.38783**	**0.16750**	0.15691	0.24632	0.32926	**0.29349**	0.33343	0.24460	0.40477
Merged	0.46763	**0.17310**	**0.23866**	**0.26765**	**0.21509**	0.13608	0.38736	0.16625	**0.16164**	**0.27901**	**0.35348**	0.18967	0.29661	0.25495	0.34478

Bold means the best performance in the case of each dataset.

**Table 6:** Concept categorization performance with *ℓ*=5 and *d*=100.

Word embeddings	AP	BLESS	Battig	ESSLI_1a	ESSLI_2b	ESSLI_2c	Ohta-10-bio-words
GloVe_W	0.21642	0.215	0.10896	0.43182	0.5	0.37778	0.41379
GloVe_C	0.22139	0.215	0.11374	0.43182	0.55	0.35555	0.40517
GloVe_Merged	0.25373	0.255	0.12043	0.43181	0.5	0.37778	0.43965
WE	0.22637	**0.29**	0.11891	0.47727	0.5	0.35556	0.38793
CE	0.23134	0.285	0.11795	0.45455	0.525	0.33333	0.41379
Merged	**0.26617**	0.275	**0.12120**	**0.5**	**0.55**	**0.4**	**0.42242**

Bold means the best performance in the case of each dataset.

**Table 7:** Concept categorization performance with *ℓ*=5 and *d*=200.

Word embeddings	AP	BLESS	Battig	ESSLI_1a	ESSLI_2b	ESSLI_2c	Ohta-10-bio-words
GloVe_W	0.22636	0.22	0.11393	0.43182	0.525	0.4	0.48275
GloVe_C	0.22388	0.23	0.11049	0.40909	0.5	0.35556	0.45689
GloVe_Merged	0.23880	0.25	0.11948	0.47727	0.525	**0.4**	0.44827
WE	0.26119	**0.33**	0.12388	**0.65909**	0.525	0.35556	0.49138
CE	0.25373	0.295	0.12235	0.56818	**0.6**	0.37778	0.48276
Merged	**0.26119**	0.305	**0.12483**	0.5	0.525	0.4	**0.49138**

Bold means the best performance in the case of each dataset.

**Table 8:** Concept categorization performance with *ℓ*=10 and *d*=100.

Word embeddings	AP	BLESS	Battig	ESSLI_1a	ESSLI_2b	ESSLI_2c	Ohta-10-bio-words
GloVe_W	0.23631	0.23	0.11489	0.43182	0.475	0.37778	0.41379
GloVe_C	0.23383	0.22	0.1158	0.43182	0.5	0.42222	0.41379
GloVe_Merged	0.25124	0.245	0.12426	**0.54545**	0.55	**0.46667**	0.45689
WE	**0.27612**	0.295	0.12177	0.47727	0.575	0.37778	0.44826
CE	0.22886	**0.32**	0.11872	0.47727	0.55	0.33333	0.43104
Merged	0.26119	0.28	**0.12732**	0.5	**0.575**	0.4	**0.48276**

Bold means the best performance in the case of each dataset.

**Table 9:** Concept categorization performance with *ℓ*=10 and *d*=200.

Word embeddings	AP	BLESS	Battig	ESSLI_1a	ESSLI_2b	ESSLI_2c	Ohta-10-bio-words
GloVe_W	0.22388	0.235	0.11871	0.43182	0.525	0.42222	0.5
GloVe_C	0.22139	0.235	0.11527	0.43182	0.525	0.37778	0.49137
GloVe_Merged	0.23383	0.275	0.12349	0.52272	**0.55**	**0.44444**	0.49137
WE	0.26368	0.285	0.12005	0.52273	0.525	0.37778	0.47414
CE	**0.26866**	0.31	**0.12388**	0.5	0.5	0.4	**0.5**
Merged	0.25871	**0.315**	0.12330	**0.65909**	0.525	0.37778	0.42241

Bold means the best performance in the case of each dataset.

**Table 10:** CNN classification performance using embeddings over the *BioText Berkeley* dataset.

Embeddings	Accuracy							
	*ℓ*=5, *d*=100		*ℓ*=5, *d*=200		*ℓ*=10, *d*=100		*ℓ*=10, *d*=200	
	Training	Validation	Training	Validation	Training	Validation	Training	Validation
GloVe_C	**0.8887**	0.8592	0.9177	0.8211	**0.8907**	**0.8592**	0.9073	0.8651
GloVe_W	0.8858	0.8563	0.9047	0.8123	0.8864	0.8334	0.9021	0.8270
GloVe_Merged	0.8487	0.8475	0.8584	0.8006	0.8493	0.8358	0.8643	0.8211
CE	0.8873	0.8646	**0.9255**	0.8323	0.8788	0.8328	0.9191	**0.8894**
WE	0.8749	**0.8652**	0.9201	**0.8423**	0.8688	0.8428	**0.9285**	0.8318
Merged	0.8507	0.8440	0.9155	0.8294	0.8516	0.8152	0.8862	0.8465

Bold means the best performance in the case of each dataset.

**Table 11:** LSTM classification performance using embeddings over the *BioText Berkeley* dataset.

Embeddings	Accuracy							
	*ℓ*=5, *d*=100		*ℓ*=5, *d*=200		*ℓ*=10, *d*=100		*ℓ*=10, *d*=200	
	Training	Validation	Training	Validation	Training	Validation	Training	Validation
GloVe_C	0.8518	0.8563	0.8474	0.8035	0.8698	**0.8822**	0.8663	0.8410
GloVe_W	0.8581	0.8492	0.8396	0.7977	0.8682	0.8651	0.8582	0.8006
GloVe_Merged	0.8230	0.8246	0.8461	0.7801	0.8376	0.8182	0.8412	0.8208
CE	**0.8880**	**0.8628**	**0.8513**	**0.8271**	0.8737	0.8765	**0.8787**	**0.8430**
WE	0.8758	0.8552	0.8474	0.8183	**0.8837**	0.8306	0.8628	0.8377
Merged	0.8321	0.8283	0.8486	0.8039	0.8482	0.8294	0.8436	0.8259

Bold means the best performance in the case of each dataset.

**Table 12:** BiLSTM classification performance using embeddings over the *BioText Berkeley* dataset.

Embeddings	Accuracy							
	*ℓ*=5, *d*=100		*ℓ*=5, *d*=200		*ℓ*=10, *d*=100		*ℓ*=10, *d*=200	
	Training	Validation	Training	Validation	Training	Validation	Training	Validation
GloVe_C	0.8463	**0.8392**	0.8310	0.7859	0.8633	0.8551	0.8689	**0.8568**
GloVe_W	0.8313	0.8122	0.8441	0.7977	0.8653	0.8534	0.8729	0.8152
GloVe_Merged	0.8266	0.8187	0.8171	0.7859	0.8389	0.8240	0.8386	0.8205
CE	0.8438	0.8337	0.8576	0.8018	**0.8753**	0.8425	0.8766	0.8501
WE	0.8431	0.8335	**0.8657**	**0.8089**	0.8616	**0.8606**	**0.8816**	0.8459
Merged	**0.8505**	0.8240	0.8318	0.7969	0.8446	0.8394	0.8468	0.8313

Bold means the best performance in the case of each dataset.

**Table 13:** CNN-LSTM classification performance using embeddings over the *BioText Berkeley* dataset.

Embeddings	Accuracy							
	*ℓ*=5, *d*=100		*ℓ*=5, *d*=200		*ℓ*=10, *d*=100		*ℓ*=10, *d*=200	
	Training	Validation	Training	Validation	Training	Validation	Training	Validation
GloVe_C	0.9177	0.8798	0.9099	0.8328	0.9134	**0.8768**	0.9167	0.8739
GloVe_W	0.9034	**0.8856**	0.8783	0.8123	0.9021	0.8768	0.9203	0.8358
GloVe_Merged	0.8897	0.8534	0.8620	0.8035	0.8676	0.8358	0.9014	0.8358
CE	**0.9202**	0.8658	0.8997	0.8501	0.8866	0.8587	0.9192	**0.8875**
WE	0.9094	0.8218	**0.9240**	0.8387	**0.9173**	0.8482	**0.9265**	0.8718
Merged	0.8984	0.8599	0.8806	**0.8603**	0.8728	0.8223	0.9175	0.8418

Bold means the best performance in the case of each dataset.

**Table 14:** CNN classification performance using embeddings over the *PubMed_20k_RCT* dataset.

Embeddings	Accuracy							
	*ℓ*=5, *d*=100		*ℓ*=5, *d*=200		*ℓ*=10, *d*=100		*ℓ*=10, *d*=200	
	Training	Validation	Training	Validation	Training	Validation	Training	Validation
GloVe_C	0.7084	0.6841	0.7381	**0.7320**	**0.7305**	0.7093	0.7087	0.7197
GloVe_W	0.7110	0.6948	0.7146	0.7148	0.7137	0.7036	0.7147	0.7264
GloVe_Merged	0.6806	0.6737	0.6779	0.6497	0.6828	0.6796	0.6868	0.6844
CE	0.7107	0.6858	**0.7451**	0.7260	0.7166	0.7128	**0.7538**	**0.7339**
WE	**0.7166**	**0.7064**	0.7389	0.7263	0.7214	**0.7180**	0.7464	0.7327
Merged	0.6998	0.6764	0.7289	0.7118	0.6993	0.6888	0.7333	0.7086

Bold means the best performance in the case of each dataset.

**Table 15:** LSTM classification performance using embeddings over the *PubMed_20k_RCT* dataset.

Embeddings	Accuracy							
	*ℓ*=5, *d*=100		*ℓ*=5, *d*=200		*ℓ*=10, *d*=100		*ℓ*=10, *d*=200	
	Training	Validation	Training	Validation	Training	Validation	Training	Validation
GloVe_C	0.7605	0.7589	**0.7826**	0.7522	0.7601	0.7583	0.7724	0.7719
GloVe_W	0.7589	0.7566	0.7708	0.7680	0.7612	0.7559	0.7726	0.7540
GloVe_Merged	0.7309	0.7295	0.7407	0.7378	0.7324	0.7201	0.7433	0.7405
CE	**0.7667**	**0.7606**	0.7785	0.7554	0.7687	**0.7596**	**0.7856**	**0.7754**
WE	0.7571	0.7559	0.7819	**0.7731**	**0.7707**	0.7587	0.7849	0.7699
Merged	0.7386	0.7297	0.7771	0.7497	0.7431	0.7397	0.7592	0.7486

Bold means the best performance in the case of each dataset.

**Table 16:** BiLSTM classification performance using embeddings over the *PubMed_20k_RCT* dataset.

Embeddings	Accuracy							
	*ℓ*=5, *d*=100		*ℓ*=5, *d*=200		*ℓ*=10, *d*=100		*ℓ*=10, *d*=200	
	Training	Validation	Training	Validation	Training	Validation	Training	Validation
GloVe_C	**0.7588**	0.7478	0.7705	0.7650	0.7593	**0.7573**	0.7706	0.7631
GloVe_W	0.7569	0.7464	0.7707	**0.7699**	0.7601	0.7470	0.7719	0.7680
GloVe_Merged	0.7306	0.7279	0.7411	0.7381	0.7328	0.7283	0.7414	0.7410
CE	0.7545	0.7362	0.7850	0.7667	0.7598	0.7561	0.7909	0.7687
WE	0.7576	**0.7481**	**0.7898**	0.7685	**0.7667**	0.7486	**0.7941**	**0.7727**
Merged	0.7326	0.7285	0.7501	0.7449	0.7396	0.7315	0.7786	0.7532

Bold means the best performance in the case of each dataset.

**Table 17:** CNN-LSTM classification performance using embeddings over the *PubMed_20k_RCT* dataset.

Embeddings	Accuracy							
	*ℓ*=5, *d*=100		*ℓ*=5, *d*=200		*ℓ*=10, *d*=100		*ℓ*=10, *d*=200	
	Training	Validation	Training	Validation	Training	Validation	Training	Validation
GloVe_C	0.7275	**0.7217**	**0.7564**	0.7497	0.7246	0.7156	0.7509	0.7340
GloVe_W	0.7233	0.7126	0.7220	0.7278	0.7275	0.7175	0.7473	0.7379
GloVe_Merged	0.7107	0.7010	0.7121	0.7207	0.7190	0.7049	0.7327	0.7231
CE	**0.7337**	0.7186	0.7515	0.7440	0.7390	0.7195	0.7908	0.7553
WE	0.7303	0.7184	0.7532	**0.7505**	**0.7418**	**0.7293**	**0.7960**	**0.7756**
Merged	0.7273	0.7094	0.7507	0.7491	0.7347	0.7109	0.7785	0.7531

Bold means the best performance in the case of each dataset.

## Data Availability

The data used to support the findings of this study are available upon reasonable request to the corresponding authors.
